# Improved Sparrow Algorithm Based on Game Predatory Mechanism and Suicide Mechanism

**DOI:** 10.1155/2022/4925416

**Published:** 2022-05-16

**Authors:** Ping Yang, Shaoqiang Yan, Donglin Zhu, Jiangpeng Wang, Fengxuan Wu, Zhe Yan, Song Yan

**Affiliations:** ^1^Xi'an Research Institute of High Technology, Xi'an, Shaanxi 710025, China; ^2^School of Information Engineering, Jiangxi University of Science and Technology, Ganzhou, Jiangxi 341000, China

## Abstract

In order to overcome the defect that sparrow search algorithm converges very fast but is easy to fall into the trap of local optimization, based on the original mechanism of sparrow algorithm, this paper proposes game predatory mechanism and suicide mechanism, which makes sparrow algorithm more in line with its biological characteristics and enhances the ability of the algorithm to get rid of the attraction of local optimization while retaining the advantages of fast convergence speed. By initializing the population with the good point set strategy, the quality of the initial population is guaranteed and the diversity of the population is enhanced. In view of the current situation that the diversity index evaluation does not consider the invalid search caused by individuals beyond the boundary in the search process, an index to measure the invalid search beyond the boundary in the search process is proposed, and the measurement of diversity index is further improved to make it more accurate. The improved algorithm is tested on six basic functions and CEC2017 test function to verify its effectiveness. Finally, the improved algorithm is applied to the three-dimensional path planning of UAV with threat area. The results show that the improved algorithm has stronger optimization performance, has strong competitiveness compared with other algorithms, and can quickly plan the effective and stable path of UAV, which improves an effective method for the application in this field and other fields.

## 1. Introduction

With the progress of modern technology, intelligent algorithms also continue to develop [1–5] and are applied to all kinds of engineering applications and real life. Comparing the swarm intelligence optimization algorithm and traditional optimization algorithm, the former is a heuristic search technology based on biological population characteristics. It has fast convergence speed, strong robustness, and high stability. With its own self-organization and adaptive characteristics, it can effectively solve complex optimization problems. The continuous development of swarm intelligence algorithm not only opens up a new world for solving various complex engineering problems but also stimulates the great research interest of scholars. Various swarm intelligence optimization algorithms appear one after another, and the family of swarm intelligence optimization algorithms has been unprecedentedly developed [6–9]. New algorithms are constantly proposed, such as naked mole-rat algorithm (NMRA) [10], firefly algorithm (FA) [11], ant lion optimizer (ALO) [12], whale optimization algorithm (WOA) [13], sine cosine algorithm (SCA) [14], crow search algorithm (CSA) [15], Harris hawks optimization (HHO) [16], slime mould algorithm (SMA) [17], hunger games search (HGS) [18], Runge–Kutta method [19], and colony predation algorithm (CPA) [20].

Inspired by sparrows' foraging behavior, predatory behavior, and antipredation behavior, a new swarm intelligence optimization algorithm, sparrow search algorithm (SSA) [21], was proposed by Xue et al. in 2020. Compared with traditional intelligent optimization algorithms, such as bat algorithm (BA) [22], grey wolf optimization (GWO) [23], and whale optimization algorithm (WOA) [13], SSA has the advantages of fast convergence, high stability, and strong robustness [24].

The algorithm has the advantage of fast convergence speed, but the global search ability is poor, the optimization results have great randomness, and it is easy to fall into the trap of local optimization. In view of this defect, many scholars have proposed different improvement strategies to improve the performance of sparrow algorithm and successfully solve many complex engineering problems [25]. In literature [26], the search mechanism of bird swarm algorithm replaces the original search mechanism, enhances the global search ability, and effectively breaks through the local limited search. Literature [27] makes full use of the current dominant individuals through the iterative local search mechanism, making the search method more diversified and the optimization accuracy more detailed. Literature [28] introduced the dimension-by-dimension lens learning mechanism to reduce the interference between dimensions and accelerate the convergence of the population. Inspired by logistic model, literature [29] proposed a new adaptive factor to dynamically control the safety threshold, which balances the ability of global search and local development of the algorithm.

The above algorithm has improved the sparrow algorithm and achieved some results, but there are still some shortcomings:

1. The improved initialization method still has some randomness, which cannot guarantee the quality of each initialization population.
2. The mechanism that the follower only pillages food with the discoverer's optimal solution does not accord with the characteristics of biological population and makes insufficient use of other optimal solutions, so it is easy to skip the global optimal solution and miss it.
3. The location update method of followers is to directly jump to the vicinity of the current optimal solution. Although this method leads to the advantage of fast convergence speed, it is also very easy to fall into local optimization. Once it cannot jump out of local optimization, it will reduce the optimization performance.

To solve the above problems, based on the summary of previous work, this paper presents an improved sparrow search algorithm based on game predatory mechanism and suicide mechanism (GPSSA), which helps to improve the shortcomings of SSA algorithm, such as fast convergence speed while being easy to fall into local optimization. This paper presents an improved sparrow search algorithm based on game predatory mechanism and suicide mechanism, which is more in line with the biological habits of sparrow population, ensures more uniform population through a good point set, makes full use of the better individuals in the population through game predatory mechanism and ensures the flexibility of search, and helps the algorithm jump out of local optimum through suicide mechanism. An invalid search index is presented for the true location of individuals beyond the boundary during the search process, which improves the defect of the original index and makes it more accurate and realistic to reflect the population diversity, exploration, and development stages in the search process. The improved GPSSA has the advantages of good initialization population quality, flexible search ability, good population diversity, and fast convergence speed. It is easy to get rid of the characteristics of local optimal attraction. The main contributions are as follows:

1. By adding good point set, the initial population is more uniform, the population is more diverse, and the quality of the initial population is guaranteed.
2. On the basis of the original mechanism, a game predatory mechanism is proposed, which makes the algorithm more in line with biological characteristics and makes the search ability of the algorithm more flexible without reducing the advantages of fast convergence speed of the original algorithm.
3. According to the unique biological characteristics of sparrows that cannot be kept in captivity, a suicide mechanism is proposed, which is to die and live afterwards, eliminate the original individuals and produce new individuals, help the algorithm increase the population diversity, and jump out of the local optimum.
4. On the basis that the original population diversity index does not consider the individuals beyond the boundary in the search process, an index to measure the invalid search of individuals beyond the boundary is proposed, and the original population diversity index is improved to make the results more accurate.
5. Six basic test functions are used for experimental simulation. The step size diagram, diversity index analysis, and development exploration stage index are used to analyze the role and effect of each strategy. The improved algorithm is compared with particle swarm optimization (PSO) [30], differential evolution (DE) [31], grey wolf optimization (GWO) algorithm [23], and sparrow search algorithm (SSA) [21] to verify its applicability.
6. CEC2017 [32, 33] is used to verify the effect of GPSSA algorithm in more complex computing environment. On the basis of the above algorithm, newer cuckoo search (CS) algorithm [34] and multistrategy serial cuckoo search (MSSCS) algorithm [35] are added for comparison and analysis to verify its superiority, and Wilcoxon rank-sum analysis, box chart, and radar sorting chart are used to verify the effectiveness of the algorithm.
7. The improved algorithm (GPSSA) is applied to a discrete problem, UAV path planning with threat [36], to help UAV quickly plan the optimal path.

## 2. Sparrow Search Algorithm

SSA is a new swarm intelligence optimization algorithm proposed by sparrows' foraging behavior, predatory behavior, and antipredatory behavior. Its bionic principle is as follows.

When the sparrow population is foraging, the individual population can be divided into discoverer, follower, and scouter. The discoverer is responsible for finding the food and leading the population to search the direction. The follower follows the discoverer to seize the food. The scouter is alert to the threat of the surrounding environment and sends a danger signal in time to remind the sparrow population to move to a safer area.

When the sparrow population does not find the existence of predators or other external threats, the search and foraging environment is safe. The discoverer can perform a wide range of search operations to guide the population to obtain higher energy. When the scouter discovers the threat of the external environment or the presence of predators, with the release of the scouter's early warning signal, the discoverer timely adjusts the search strategy and quickly approaches the safe area. Therefore, the location update formula for the discoverer to guide the population foraging is set as follows:

(1) $$\begin{array}{c} X_{i,j}^{t+1}=\left\{\begin{array}{cc} X_{i,j}^{t}\cdot \text{exp}\left(\frac{-i}{\alpha \cdot M}\right), & R_{2}<\text{ST},\\ X_{i,j}^{t}+Q\cdot L, & R_{2}\geq \text{ST}. \end{array}\right.. \end{array}$$

In the above formula, *X*_*i,j*_ represents the current position of the *i-*th sparrow in the *j-*th dimension. *M* is the maximum number of iterations. *t* represents the current number of iterations. *R*_2_ represents an early warning value belonging to [0, 1]. *α* is a random number belonging to [0, 1]. ST is the security threshold belonging to [0.5,1]. *L* stands for a 1 × *d* matrix, and all elements in the matrix are 1. *Q* is a random number subject to normal distribution.

When the followers follow the discoverers without food, they are very hungry and have low energy, so they need to fly to other places to find food to improve their energy. When the followers follow the discoverer to get food, they only need to find a place near the best position of the sparrow population for foraging. Based on this, the location update formula of the participant is set as follows:

(2) $$\begin{array}{c} X_{i,j}^{t+1}=\left\{\begin{array}{cc} Q\cdot \;\exp\left(\frac{X_{\text{worst}}^{t}-X_{i,j}^{t}}{i^{2}}\right), & i>\frac{n}{2},\\ X_{P}^{t+1}+\left|X_{i,j}^{t}-X_{P}^{t+1}\right|\cdot A^{+}\cdot L, & \text{otherwise.} \end{array}\right. \end{array}$$

In the above formula, *X*_*p*_ is the best position currently occupied by the discoverer, and *X*_worst_ represents the worst position. *A* is a 1 × *d* matrix with only 1 or −1 elements, where *A*^+^ = *A*^T^(*AA*^T^)^−1^.

When *i* *>* *n*/2, it means that the *i*-th follower with low fitness does not get food, is in a very hungry state, and needs to fly to other places to find food. When *i* *≤* *n*/2, followers will compete for food with the discoverer who finds the most food (with the best fitness), so as to improve their energy.

When the scouter is at the edge of sparrow population, it is very vulnerable to predator attack or other external environment threats, so the scouter needs to quickly move closer to the global optimal position to reduce the threat. When the scouters are in the middle of the population, if they are aware of the danger information, they will timely get close to other sparrows, so as to reduce the risk of being attacked or preyed on. Therefore, the scouter position update formula is set as follows:

(3) $$\begin{array}{c} X_{i,j}^{t+1}=\left\{\begin{array}{cc} X_{\text{best}}^{t}+\beta \cdot \left|X_{i,j}^{t}-X_{\text{best}}^{t}\right|, & f_{i}\neq f_{g},\\ X_{i,j}^{t}+K\cdot \left(\frac{\left|X_{i,j}^{t}-X_{\text{worst}}^{t}\right|}{\left(f_{i}-f_{w}\right)+\varepsilon }\right), & f_{i}=f_{g}. \end{array}\right. \end{array}$$

*X*_best_ represents the global optimal position of the current population. *β* is responsible for controlling the step size parameter, which is a random number subject to standard normal distribution. *K* is responsible for controlling the moving direction and step of sparrow, which is a random number belonging to [−1, 1]. *f*_*i*_ is the fitness value of the current *i*-th sparrow individual. *f*_*g*_ and *f*_*w*_, respectively, represent the best and worst fitness values of the current population. *ε* is a minimal real number.

## 3. Improved Sparrow Algorithm Based on Game Predatory Mechanism and Suicide Mechanism (GPSSA)

### 3.1. Good Point Set

The good point set was proposed by Chinese mathematicians Hua and Wang [37], and its principle is as follows: let *G*_*S*_ be the unit cube in *s*-dimensional Euclidean space, and if *r* ∈ *G*_*s*_, the form is

(4) $$\begin{array}{c} P_{n}\left(k\right)=\left\{\left(\left\{r_{1}^{\left(n\right)}\cdot k\right\},\left\{r_{2}^{\left(n\right)}\cdot k\right\},\ldots \left\{r_{s}^{\left(n\right)}\cdot k\right\}\right),1\leq k\leq n\right\}. \end{array}$$

If the deviation *φ*(*n*) satisfies *φ*(*n*)=*C*(*r*, *ε*)*n*^−1+*ε*^, *ε* is any positive number, where *C*(*r*, *ε*)*n*^−1+*ε*^ is a constant only related to *r* and *ε*. *P*_*n*_(*k*) is a good point set and *r* is a good point. {*r*_*s*_^(*n*)^ · *k*} represents the decimal part, *n* represents the number of points, and *r*={2  cos(2*πk*/*p*), 1 ≤ *k* ≤ *s*} , where *p* is the minimum prime number satisfying (*p* − 3)/2 ≥ *s*. Map it to the search space [34] as

(5) $$\begin{array}{c} x_{i}\left(j\right)=\left(ub_{j}-lb_{j}\right)\cdot \left\{r_{j}^{\left(i\right)}\cdot k\right\}+lb_{j}, \end{array}$$

where *ub*_*j*_ and *lb*_*j*_ represent the upper and lower bounds of the *j*-th dimension, respectively.

Figure 1(a) shows a randomly generated initial population distribution map when the good point set is in [0, 1], the number of populations is 500, and the dimension is 1. Figure 1(b)shows the frequency distribution histogram of good point set and tent chaotic map [35] under the above conditions. It can be seen that the good point integration is evenly distributed, and the initialization effect is better than that of tent chaotic map. In the initialization process, the good point set has a more uniform population, which can increase the diversity of the population and help to eliminate the attraction of the local optimal solution.

### 3.2. Game Predatory Mechanism

The followers in sparrow algorithm have a predatory mechanism; that is, the followers directly jump to the vicinity of the optimal location of the discoverer to compete for food. However, the food in the best position of the discoverer is not endless, and it is impossible to meet the food needs of a large number of followers, which is also inconsistent with the laws of nature. Therefore, based on the game theory, this paper proposes a game predator mechanism; that is, the predatory mechanism of followers and discoverers is regarded as a game process. When *i* < *N*/2, it is stipulated that the food found by each discoverer can only meet the needs of limited participants, and the amount of food found is determined by its fitness value. The top followers will give priority to those who find the most food to grab food. In order to obtain food and avoid hunger, the lower ranked participants will choose the discoverer who finds less food to eat, as shown in Figure 2(a). It is worth noting that, for the mechanism when *i* *>* *N*/2, the followers obtain food and forage alone is retained, as shown in Figure 2(b).

It is found from (2) that when *i* *≤* *N*/2, the followers will grab food after the discoverers. Therefore, there are *R* followers who directly jump to the vicinity of the discoverer who finds the most food and grab food, where *R*=*N*/2 − PD · *N* and PD is the proportion of discoverers.

Assuming that the food found by each discoverer is limited, the food in the optimal location of the discoverer cannot meet the food needs of a large number of followers, and the followers participating in the predator mechanism will grab food from different discoverers because of the shortage of food. At this time, it is a game process, and the followers will choose the discoverer who is most favorable to them to grab food. There are two steps in the game predatory mechanism: one is to count the food quantity of the discoverer, and the other is to make game selection to select the most beneficial discoverer for oneself as follows.

#### 3.2.1. Food Quantity Statistics of Discoverer

Individuals with lower fitness are considered to be better choices. The lower the fitness of the discoverer's location is, the more food is found, and the number of discoverers is PD · *N*. *D*_*z*_ represents the *z*-th discoverer. Then the quantity *G* of food found by the *z*-th discoverer can be expressed as

(6) $$\begin{array}{c} G_{z}=\frac{1}{f\left(D_{z}\right)},\;z=1,2,\ldots ,\text{PD}\cdot N. \end{array}$$

#### 3.2.2. Game Choice

When *J*_*z*_ followers compete for food with the *z*-th discoverer, the subsequent followers will choose to compete for food with the *z* + 1-th discoverer because of the game mechanism, and so on. *F*_*j*_ represents the *j*-th follower. *J*_*z*_ is determined by the ratio *p*_*z*_ of the quantity *G*_*z*_ of food found by the *z*-th discoverer to the total quantity. The specific principle is as follows:

(7) $$\begin{array}{c} p_{z}=\frac{G_{z}}{\sum_{z=1}^{\text{PD}\cdot N}G_{z}}, \end{array}$$

(8) $$\begin{array}{c} J_{z}=\text{round}\left(p_{z}\cdot R\right). \end{array}$$

At this time, the relationship between each follower in the game predatory mechanism and its predatory discoverer is as follows:

(9) $$\begin{array}{c} D_{1}\left\{\begin{array}{c} F_{1}\\ F_{2}\\ \cdots \\ F_{J_{1}} \end{array}\right.,D_{2}\left\{\begin{array}{c} F_{J_{1}+1}\\ F_{J_{1}+2}\\ \cdots \\ F_{J_{1}+J_{2}} \end{array}\right.,\cdots ,D_{P\;D\cdot N}\left\{\begin{array}{c} F_{J_{1}+J_{2}+\cdots +J_{\text{PD}\cdot N-1}+1},\\ F_{J_{1}+J_{2}+\cdots +J_{\text{PD}\cdot N-1}+2},\\ \cdots \\ F_{J_{1}+J_{2}+\cdots +J_{\text{PD}\cdot N}}. \end{array}\right.. \end{array}$$

Therefore, the location update formula of the improved followers is as follows:

(10) $$\begin{array}{c} X_{i,j}^{t+1}=\left\{\begin{array}{cc} Q\cdot \text{exp}\left(\frac{X_{\text{worst}}^{t}-X_{i,j}^{t}}{i^{2}}\right), & i>\frac{N}{2},\\ D_{z,j}^{t+1}+\left|X_{i,j}^{t}-D_{z,j}^{t+1}\right|\cdot A^{+}\cdot L, & \text{otherwise.} \end{array}\right. \end{array}$$

### 3.3. Suicide Mechanism

Sparrows mostly live in places where human beings live. They are very lively, bold, and approachable, but they are very vigilant. Sparrows are very proud birds. They live on people, but they do not want to be kept in captivity. If they do not have freedom, they would rather starve to death [38]. Therefore, this paper adds a suicide mechanism to the original mechanism of the sparrow search algorithm. *t*_*i*_ represents the number of iterations in which the individual's position is not updated. When the individual in the population exceeds the number of dangerous iterations *T*_*c*_ and does not update the position, it is considered that the sparrow is in an imprisoned state. At this time, the sparrow will go on hunger strike and commit suicide. At this time, we abandon the sparrow individual and generate a new sparrow individual, which helps the algorithm jump out of the local optimum. This process can be expressed by an old Chinese saying: “die and come back,” and its position is updated as follows:

(11) $$\begin{array}{c} X_{i,j}^{t+1}=\left\{\begin{array}{cc} X_{i,j}^{t}+X_{i,j}^{t}\cdot \text{randn}\left(\;\right), & t_{i}\geq T_{c},\\ X_{i,j}^{t}, & \text{otherwise.} \end{array}\right. \end{array}$$

### 3.4. GPSSA Algorithm Flow

### 3.5. Time Complexity Analysis

According to the number of populations, iteration times, and dimensions of SSA algorithm, we can easily know that the time complexity of original SSA algorithm is O (*P·M·D*). Firstly, GPSSA algorithm is improved on the basis of SSA algorithm; GPSSA has the same structure as the original algorithm and does not increase the number of cycles. Secondly, the good point set strategy replaces the original method of randomly initializing the population, but the time complexity does not increase. The game predatory mechanism only changes the way to approach the current optimal solution and further approaches the suboptimal solution to prevent the omission of the suboptimal solution, which also does not increase the time complexity. The suicide mechanism adopts greedy strategy, which increases the complexity of the searcher's algorithm to a certain extent. Only a few individuals in the population increase the complexity of the algorithm but not the order of magnitude of the entire algorithm. To sum up, we can get that the time complexity of GPSSA is still O(*P·M·D*).

## 4. Exploration and Exploitation Stage and Population Diversity

Literature [39] proposes a theoretical system to evaluate the algorithm's exploration and exploitation stage and population diversity by using the differences between individual dimensions of the population. On the basis of the above, literature [40] uses the median that can better reflect the population center instead of the average to calculate the dimensional diversity, and the effect is more accurate. The calculation formula is shown in (12). When the population diverges, it indicates that it is in the exploration stage, and the calculation formula is shown in (12). When the population gathers, it indicates that it is in the exploitation stage, and the calculation formula is shown in the following equation:

(12) $$\begin{array}{c} {\text{Div}}_{j}=\frac{\sum_{i=1}^{N}\left|\text{median}\left(x_{j}\right)-x_{i,j}\right|}{N},\\ \text{Div}=\frac{\sum_{j=1}^{D}{\text{Div}}_{j}}{D},\\ X_{\text{pl}}=\frac{\text{Div}}{{\text{Div}}_{\text{max}}},\\ X_{\text{pt}}=\frac{\left|\text{Div}-{\text{Div}}_{\text{max}}\right|}{{\text{Div}}_{\text{max}}}, \end{array}$$

where median(*x*_*j*_) represents the median of the *j*-th dimension of the whole population, *x*_*i*,*j*_ represents the *j*-th dimension of the *i*-th individual, Div_*j*_ represents the diversity of the *j*-th dimension, Div represents the diversity of the whole population, and Div_max_ represents the maximum population diversity in the iterative process. In the search process, *X*_pl_ and *X*_pt_ represent the percentages of exploration and exploitation stages, respectively.

### 4.1. Invalid Search Indicator

The above method does not take into account the fact that when an individual exceeds the boundary in the search process, the individual beyond the boundary will be corrected to the boundary in the next iteration. Therefore, the position beyond the boundary is invalid, and the diversity of the population is also invalid or inaccurate. Therefore, this paper proposes an index Inv to evaluate the invalid search beyond the boundary of the algorithm, which is used to describe the ability of invalid search in the *t*-th iteration of the algorithm. The specific expression is as follows:

(13) $$\begin{array}{c} \text{Inv}=\frac{1}{N\cdot D}\sum_{i=1}^{N}\sum_{j=1}^{D}\text{max}\left(\left|\text{min}\left(X_{i,j}^{t}-lb_{j},0\right)\right|,\left|\text{min}\left(ub_{j}-X_{i,j}^{t},0\right)\right|\right), \end{array}$$

where |min(*X*_*i*,*j*_^*t*^ − lb, 0)| and |min(ub − *X*_*i*,*j*_^*t*^, 0)| are used to determine the distance values of *lb* and *ub* beyond the boundary. If it does not exceed the boundary, the value is 0. max(|min(*X*_*i*,*j*_^*t*^ − lb, 0)|, |min(ub − *X*_*i*,*j*_^*t*^, 0)|) is used to calculate the distance beyond the boundary. It is easy to know that one of the two must be 0, because it can only exceed one side of the boundary. The smaller the value, the stronger the ability of the algorithm to search effectively.

### 4.2. Improved Exploration and Exploitation Stage and Population Diversity

If the above indexes for evaluating the invalid search ability are brought into the original index system, more accurate indexes of population diversity and exploration and exploitation stage can be obtained. For individuals beyond the boundary in the search process, the strategy of modifying to the boundary will be adopted in the next iteration, so the boundary position is the real position of individuals beyond the search boundary. Since the individuals beyond the boundary do not affect the selection of the median, the improved formula is as follows:

(14) $$\begin{array}{c} {\text{Div}}^{\prime }=\text{Div}-\text{Inv,} \end{array}$$

(15) $$\begin{array}{c} X_{\text{pl}}^{\prime }=\frac{{\text{Div}}^{\prime }}{{\text{Div}}_{\text{max}}^{\prime }}, \end{array}$$

(16) $$\begin{array}{c} X_{\text{pt}}^{\prime }=\frac{\left|{\text{Div}}^{\prime }-{\text{Div}}_{\text{max}}^{\prime }\right|}{{\text{Div}}_{\text{max}}^{\prime }}. \end{array}$$

## 5. Experimental Simulation of Basic Test Function

In this paper, six basic test functions are selected to verify the performance of GPSSA algorithm and compared with other heuristic algorithms, such as PSO, DE, GWO, SSA, and GPSSA. The specific parameter settings are shown in Table 1. F1–F3 are high-dimensional single peak benchmark functions, F4-F5 are high-dimensional multipeak benchmark functions, and F6 is low-dimensional multipeak benchmark function. The test function information is shown in Table 2, and the parameter space is shown in Figure 3.

Figure 4 shows the initial population of the above algorithm and the step size update after only one iteration, in which the objective function is F1 and the number of populations is 100. The red cross in the figure is the location of the optimal solution. As can be seen from the figure, the step amplitude of PSO update is small, and the step amplitude of DE and GWO is large. However, the optimal solution found after initializing the population is not fully utilized by DE and GWO, resulting in blind search. Because of the influence of the discoverer-follower mechanism, most of the population individuals converge near the optimal solution, which is also the main reason why the SSA algorithm has the advantage of fast convergence speed. However, it is also easy to fall into the dilemma of local optimization, and it can be seen from the figure that the initial population of GPSSA is more uniform due to the influence of good point set strategy. Due to the game predatory mechanism, some followers will approach the current suboptimal solution to prevent missing the better solution and falling into the local optimum.

Figure 5 shows the comparison of the effects of the three strategies proposed in this paper. Set the population number to 30 and the number of iterations to 500, and select F1 as the objective function, where (a) is 30 dimensions and (b) is 100 dimensions. SSA is the original algorithm; SSA1, SSA2, and SSA3 are the improved algorithms with good point set strategy, game predatory mechanism, and suicide mechanism separately added to SSA; and GPSSA is the improved algorithm with three strategies added. As can be seen from the above figure, the addition of these three strategies can improve the performance of SSA algorithm to a certain extent. At 30 dimensions, SSA1 and SSA2 are better; at 100 dimensions, the effect of SSA2 and SSA3 is more obvious when the dimension increases, but SSA1 has no significant change. The effect of GPSSA is better than that of a single strategy, which shows that the good point set strategy, game predatory mechanism, and suicide mechanism all have a good improvement effect on the original algorithm.

Table 3 shows the comparison of optimization effects of each algorithm running independently for 30 times, in which the population size is 30, the maximum number of iterations of each algorithm is 500, and the best value of each index is displayed in bold. Finally, the average value is used to sort each algorithm (if the average value is equal, consider the standard deviation). It can be seen from the table that GPSSA shows excellent optimization performance. GPSSA has found the optimal value in F1–F6, indicating that GPSSA has good optimization ability; each index is almost the best in all algorithms, and the comprehensive ranking is also the first, indicating that GPSSA has good optimization accuracy and stability. Except for F5, the results of GPSSA and SSA are the same. In other functions, GPSSA has found a better solution than SSA, indicating that GPSSA algorithm has stronger optimization performance than the original algorithm.

Figure 6 shows the convergence diagram of each algorithm in the above function. GPSSA has faster convergence speed and better optimization accuracy than SSA. In F1 and F2, the convergence rate of GPSSA is very stable, almost in a straight line, and there is no cliff decline like SSA, indicating that the game predatory mechanism has stronger and more stable optimization ability than the original SSA predatory mechanism. In F3 and F4, SSA falls into the local optimum, while GPSSA will regenerate new individuals to jump out of the local optimum after stopping updating due to the suicide mechanism. In F5, although both SSA and GPSSA find the optimal solution, the convergence speed of GPSSA is faster. In F6, both SSA and GPSSA find the optimal solution after falling into the local optimum, which shows that the original SSA algorithm also has a certain ability to jump out of the local optimum, but GPSSA has a stronger ability to jump out of the local optimum.

Figure 7 shows the invalid search index of each algorithm obtained according to formula (13), which is used to represent the index of invalid search caused by exceeding the boundary in the search process. The change trend of this index is mainly related to the update mechanism of the algorithm location. For example, the population will continue to converge in the search process of PSO, DE, and GWO algorithms, so it will continue to decrease with the number of iterations. Although SSA and GPSSA will also converge and converge faster, due to the antipredation behavior in the algorithm, some population individuals will continue to escape the current position and will not be reduced by the number of iterations, such as F3 and F6. F1, F2, F4, and F5 are not affected by the update step size and boundary size.

Because an individual experiences the phenomenon of exceeding the boundary in the search process and the individual is corrected to the boundary in the next iteration update, the boundary position is the real position of the individual exceeding the boundary in the search process. The improved diversity index removes such effects and the results will be more accurate.  Figure 8 shows the population diversity calculated according to the improved formula (14). It can be seen from Figure 8 that the diversity of PSO, DE, and GWO algorithms will decrease with the number of iterations due to the continuous convergence of population individuals, and the decline speed of PSO is the slowest. SSA and GPSS algorithms decline faster, but because the vigilant mechanism continues to escape from the current position, it will not fall to 0, but it will continue to fluctuate to maintain population diversity and prevent falling into local optimization. Combined with Figure 6, we can find that when SSA and GPSSA no longer converge (when the convergence curve level or no longer decreases), the population diversity will suddenly rise due to the antipredation behavior, which helps the algorithm jump out of the local optimum. At the same time, due to the suicide mechanism, GPSSA will think that it is in an imprisoned state at this time and then commit suicide to produce new individuals, which will have better population diversity compared to the SSA algorithm.

According to equations (15) and (16), Figure 9 shows the exploration-exploitation ratio of each algorithm in six functions, where (a), (b), (c), (d), (e), and (f) are the development exploration ratio under F1, F2, F3, F4, F5, and F6, respectively. As can be seen from the figure, PSO, DE, and GWO algorithms all change from exploration stage to exploitation stage with the number of iterations, and the exploitation percentage increases and the exploration percentage decreases. SSA and GPSS algorithms enter the development stage after very few iterations because of their fast convergence speed. Combined with Figure 6, we can find that when SSA and GPSSA are no longer convergent, the development percentage continues to decline, the exploration percentage increases, and the development stage changes to the exploration stage to prevent them from falling into local optimization. Due to the addition of three strategies, GPSSA has better search ability and the ability to jump out of local optimization, which leads GPSSA to find the optimal solution earlier, end the exploitation stage, and then enter the exploration stage.

## 6. CEC2017 Test

In order to further verify the generality of the algorithm, the algorithm is tested on CEC2017 test function [41]. Due to the defects of F2 function, this paper will not test. The number of dimensions is 30, the number of individuals is 100, the number of evaluations is set to 10000 ∗ dim, and the algorithm parameters remain unchanged. After 30 independent runs, the average value and standard deviation of each algorithm are calculated according to the results and finally sorted. The best value for each index is displayed in bold. The specific test results are shown in Table 4.

The results in Table 4 show that the average value of GPSSA algorithm is the best value among all algorithms in F1, F5, F8, F9, f13, F14, F15, F16, F17, F19, F21, F23, F24, F26, F28, and F29 functions, which shows that GPSSA algorithm has good optimization ability and accuracy. The average ranking of GPSSA is 2.28, followed by PSO (2.97), MSSCS (2.93), CS (3.59), DE (4.76), SSA (5.48), and GWO (6.00). The SSA algorithm does not perform well in more complex CEC217. Only due to GWO, it shows that the optimization ability of the original algorithm decreases in more complex optimization problems, while the improved GPSSA is more suitable for complex optimization problems due to the improvement of mechanism.

Figure 10 shows a radar chart made according to the algorithm ranking. The higher the ranking is, the closer it is to the radar center. It can be seen that more than half of GPSSA functions are closest to the radar center, and the enclosed area is the smallest. According to the 30 times' optimal results, all algorithms conduct Wilcoxon rank-sum test for GPSSA, and the results are shown in Table 5. When the value is greater than 0.05, it can be considered that there is no significant difference between the two; otherwise, it is considered that there is a significant difference between the two, where “+” and “−” mean greater than and less than 0.05, respectively. Only a few values in the results are greater than 0.05, indicating that GPSSA algorithm is significantly different from other algorithms.  Figure 11 shows the selected six groups of box graphs, in which the box graph of GPSSA has a shorter length than other algorithms, indicating that GPSSA algorithm has strong optimization performance and stability. The results show that the optimization performance of GPSSA is better than that of SSA, and the optimization performances of PSO and MSSCS are also better.

In the SSA algorithm, when the participants in the population move closer to the discoverer, they jump directly to the current optimal solution instead of moving slowly to the current optimal solution, so the result of SSA is very poor. This problem leads to a large range of individual update steps of the population in SSA algorithm, which accelerates the convergence of the algorithm, but it is easy to miss the high-quality solution. GPSSA algorithm adopts an improved strategy to make up for this disadvantage, which makes the initial population more uniform, makes full use of other better solutions or generates new solutions, increases the population diversity, makes the search method more flexible, and greatly reduces the loss of population diversity. In general, GPSSA algorithm retains the advantage of fast convergence speed of the original algorithm, has good universality and optimization performance, and has strong competitiveness compared with other algorithms.

## 7. UAV Path Planning

UAV path planning problem [42] is an optimization problem where UAV uses terrain as cover to effectively avoid various threats, so as to improve the survivability of aircraft and quickly reach the destination. Aiming at the problem of UAV path planning, several methods such as graph theory search, element decomposition, potential field, and natural heuristic algorithm are proposed in the literature [43–45]. However, with the more and more complex tasks undertaken by UAV, the uncertainty of its flight environment, and the higher requirements for track planning, the superiority of swarm intelligence algorithm in solving complex problems makes more and more scholars apply swarm intelligence algorithm to this field. To solve the UAV track planning problem, it is necessary to establish an appropriate fitness function and consider various constraints affecting the track quality. The static global 3D track planning model mainly includes cost function and constraint function.

### 7.1. Flight Path Cost

In the actual combat mission, the fuel carried by UAV is limited, the track length can reflect the fuel consumption, and *L*_*i*_ is the track length of the *i*-th segment. That is, UAV flight fuel consumption cost can be expressed as track length:

(17) $$\begin{array}{c} f_{\text{path}}=\sum_{i=1}^{N}L_{i}. \end{array}$$

### 7.2. Flight Altitude Change Cost

In order to avoid radar search and prevent collision with mountains or other obstacles, the UAV must raise or lower the height, but repeated lifting and lowering will also endanger the safety of the UAV. The variance of track altitude change can describe the stability of flight altitude. As the cost of altitude change, it can be expressed as

(18) $$\begin{array}{c} f_{\text{height}}=\frac{\sum_{i=1}^{N}{\left(z_{i}-\left(1/N\right)\sum_{i=1}^{N}z_{i}\right)}^{2}}{N}. \end{array}$$

### 7.3. Smoothing Cost

In the flight process, the larger the deflection angle is, the more unstable the flight state of the UAV is and the less smooth the flight path is. Therefore, the smoothing cost is added to increase the stability and smoothness of UAV track, and the smoothing cost is expressed by the change degree of deflection angle *δ*. The function is set as follows:

(19) $$\begin{array}{c} f_{\text{smooth}}=\sum_{i=1}^{N}\left|\delta_{i}-\delta_{i-1}\right|. \end{array}$$

### 7.4. Integrated Threat Constraints

UAV encounters enemy air defense system when it passes through enemy areas, including detection radar, antiaircraft artillery, and ground-to-air missile. The above threats are approximated as a cylindrical area in three-dimensional plane, and the detection or attack range is used as its radius *R*. The current track segment *L*_*i*_ is divided into five segments, *M* represents the comprehensive threat, *k*_*M*_ represents the *k*-th comprehensive threat, *R*_*k*_*M*__ represents the radius of the current threat, and *d*_*k*,*i*_ represents the distance from the current threat point to each of the five equal segments. The threat cost of the current synthetic threat point to the track segment is shown in Figure 12, and its threat constraint function is

(20) $$\begin{array}{c} \text{Constraint}=\sum_{i=1}^{5N}\sum_{k_{M}=1}^{n_{M}}\max\left(\frac{R_{k_{M}}-d_{k_{M},i}}{R_{k_{M}}},0\right). \end{array}$$

*η* is a penalty function, and the trajectory planning objective function in this paper is

(21) $$\begin{array}{c} \text{min}\left(f_{\text{cost}}\right)=\omega_{1}\cdot f_{\text{path}}+\omega_{2}\cdot f_{\text{height}}+\omega_{3}\cdot f_{\text{smooth}}+\eta \cdot \text{Constraint.} \end{array}$$

In this paper, the cubic B-spline method is used to ensure better curve smoothness for UAV track smoothing. The spline curve generated during track smoothing is determined by four adjacent control points. By reducing the dependence of track smoothing on each operating point, the smoothed track is more effective, as shown in Figure 13.

### 7.5. Track Coding

An individual in a population is defined as a path connected by multiple track points, *S*_*i*_=[*s*_*x*1_, *s*_*y*1_, *s*_*z*1_, *s*_*x*2_,……*s*_xn_, *s*_yn_, *s*_zn_], in which every 3 coordinates constitute a track point in three dimensions, a total of *N* track points, and a dimension of 3 ∗ *n* for each individual.

### 7.6. Experimental Simulation

This paper establishes a three-dimensional mountain terrain using a 100 km × 150 km × 3 km digital elevation map as shown in Figure 14. There are five nonflight zones for the composite threat, with the center coordinates of (20,45), (40,75), (60,30), (80,65), and (100,30) and a radius of 15. The starting and ending coordinates are (10,90, 1.1) and (130, 10, 1.1).

*η*=10^7^, *ω*_1_=0.5, *ω*_2_=0.3, and *ω*_3_=0.2 are set. The cubic B-spline method is used to ensure better curve smoothness for UAV track smoothing.

This paper runs 20 times, with 10 track nodes , 30 dimensions, maximum number of iterations of 200, and a population of 100. The experimental results are shown in Table 6. Path planning with threats is shown in Figure 15. Top view of path planning contour is shown in Figure 16, and target function convergence is shown in Figure 17.

Combining Figures 15–17, it can be seen that SSA is trapped in a local optimum and cannot jump out. GPSSA algorithm can quickly avoid the constraints of threat area and complete path planning, and the path planning is optimal, with faster convergence speed and better accuracy. From the results in Table 6, the four indicators of GPSSA are all optimal, indicating that they have strong optimization ability and stability. The good algorithm performance of GPSSA is verified, which can quickly and accurately get rid of the constraints of threat areas and complete the unmanned aircraft path planning. This helps the unmanned aircraft path static planning to have shorter time, better path planning, and better stability.

## 8. Conclusions

In this paper, game predatory mechanism and suicide mechanism are proposed to improve sparrow search algorithm, which is more in line with the biological habits of sparrow population, ensures more uniform population through a good point set, makes full use of the better individuals in the population through game predatory mechanism and ensures the flexibility of search, and helps the algorithm get rid of the trap of local optimization through suicide mechanism. An invalid search index is presented for the true location of individuals beyond the boundary during the search process, which improves the defect of the original index and makes it more accurate and realistic to reflect the population diversity, exploration, and development stages in the search process. By comparing the basic test functions and CEC2017 with other heuristic algorithms, it is proved that GPSSA has good optimization performance and effectively improves the shortcomings of poor initial population quality, poor utilization of the current better solution, and poor ability to jump out of local optimal. It also strengthens the ability of the original algorithm to get rid of local optimal attraction while retaining the advantages of fast convergence. Through the UAV path planning simulation, the effectiveness and superiority of GPSSA are verified. Using the advantages of rapid convergence and strong optimization performance of GPSSA, it helps to quickly plan the better path. It provides a new method for the research of this kind of field and provides a good case for the research of this algorithm in other fields.

In the future, we will try to integrate with PSO and other heuristic algorithms and combine the advantages of these two algorithms to improve their poor global search ability, further improve the search performance, and better apply them to more practical problems.

## Figures and Tables

**Figure 1:** Distribution of good point set.

**Figure 2:** Principle of game grabbing mechanism.

**Figure 3:** Parameter space of function.

**Figure 4:** Algorithm step diagram.

**Figure 5:** Strategy effect comparison.

**Figure 6:** Convergence diagram of each algorithm.

**Figure 7:** Invalid search of each algorithm.

**Figure 8:** Diversity of each algorithm.

**Figure 9:** Exploration-exploitation percentage of each algorithm.

**Figure 10:** Ranking radar chart.

**Figure 11:** Box diagram of each algorithm.

**Figure 12:** Threat principle.

**Figure 13:** Cubic B-spline principle.

**Figure 14:** Original map.

**Figure 15:** Path planning with threats.

**Figure 16:** Top view of path planning contour.

**Figure 17:** Objective function convergence graph.

**Algorithm 1:** The framework of the GPSSA.

**Table 1:** Parameter settings.

Algorithm	PSO	DE	GWO	CS	MSSCS	SSA	GPSSA
Parameter	*c*1 = 2	CR = 0.2	*a* = (2 ⟶ 0)	*α* = 0.01	*α* = 0.01	SD = 0.2	*SD* = 0.2
	*c*2 = 2				*β* = 1.5		PD = 0.2
	*W*_min_ = 0.2	*F*_min_ = 0.2		*β* = 1.5	Pa = 0.25	PD = 0.2	ST = 0.8
					*c* = 0.2		
	*W*_max_ = 0.9	*F*_max_ = 0.8		*Pa* = 0.25	*PA*_max_ = 0.35	*ST* = 0.8	*Tc* = *M*/20
					*PA*_min_ = 0.25		

**Table 2:** Basic test function.

Function	Dimensions	Interval	Min
*F*_1_(*x*)=∑_*i*=1_^*n*^*x*_*i*_^2^	30/100	[−100, 100]	0
*F*_2_(*x*)=∑_*i*=1_^*n*^|*x*_*i*_|+∏_*i*=1_^*n*^|*x*_*i*_|	30	[−100, 100]	0
*F*_3_(*x*)=∑_*i*=1_^*n*^ix_*i*_^4^+random[0，1)	30	[−1.28, 1.28]	0
$F_{4}\left(x\right)=\sum_{i=1}^{n}-x_{i}\text{sin}\left(\sqrt{\left|x_{i}\right|}\right)$	30	[−500, 500]	−418.98 ∗ dim
*F*_5_(*x*)=∑_*i*=1_^*n*^[*x*_*i*_^2^ − 10 cos(2*πx*_*i*_)+10]	30	[−5.12, 5.12]	0
*F*_6_(*x*)=∑_*i*=1_^7^[(*X* − *a*_*i*_)(*X* − *a*_*i*_)^*T*^+*c*_*i*_]^−1^	4	[0, 10]	−10.4029

**Table 3:** Comparison table of optimization effect.

	Index	PSO	DE	GWO	SSA	GPSSA
F1	Best	8.93*E − *06	2.48*E + *01	6.31*E − *28	**0.00*E + *00**	**0.00*E* + 00**
	Worst	8.36*E − *04	7.54*E + *04	4.66*E − *25	1.37*E − *67	**0.00*E* + 00**
	Ave	1.63*E − *04	3.72*E + *04	5.25*E − *26	4.58*E − *69	**0.00*E* + 00**
	Std	2.13*E − *04	2.08*E + *04	1.13*E − *25	2.51*E − *68	**0.00*E* + 00**
	Rank	4	5	3	2	1

F2	Best	4.10*E − *03	5.61*E + *00	1.47*E − *16	**0.00*E + *00**	**0.00*E* + 00**
	Worst	2.71*E − *01	3.71*E + *13	1.61*E − *15	3.45*E − *40	**0.00*E* + 00**
	Ave	4.03*E − *02	1.28*E + *12	6.19*E − *16	1.15*E − *41	**0.00*E* + 00**
	Std	5.51*E − *02	6.77*E + *12	3.56*E − *16	6.30*E − *41	**0.00*E* + 00**
	Rank	4	5	3	2	1

F3	Best	6.02*E − *02	1.93*E − *03	5.47*E − *04	5.86*E − *06	**3.90E* − *06**
	Worst	3.15*E − *01	1.64*E + *02	7.20*E − *03	1.28*E − *03	**2.47E* − *04**
	Ave	1.63*E − *01	4.72*E + *01	1.93*E − *03	2.86*E − *04	**5.88E* − *05**
	Std	6.39*E − *02	5.11*E + *01	1.52*E − *03	3.05*E − *04	**5.21E* − *05**
	Rank	4	5	3	2	1

F4	Best	−7.10*E + *03	−1.13*E + *04	−7.18*E + *03	−**1.26*E + *04**	−**1.26*E* + 04**
	Worst	−3.07*E + *03	−1.61*E + *03	−3.05*E + *03	−5.56*E + *03	−**1.03*E* + 04**
	Ave	−5.37*E + *03	−4.73*E + *03	−5.62*E + *03	−9.83*E + *03	−**1.21*E* + 04**
	Std	1.12*E + *03	2.25*E + *03	1.09*E + *03	2.34*E + *03	**6.38*E* + 02**
	Rank	4	5	3	2	1

F5	Best	3.59*E + *01	6.24*E + *01	5.68*E − *14	**0.00*E + *00**	**0.00*E* + 00**
	Worst	9.06*E + *01	4.45*E + *02	7.83*E + *00	**0.00*E + *00**	**0.00*E* + 00**
	Ave	5.76*E + *01	3.11*E + *02	9.05*E − *01	**0.00*E + *00**	**0.00*E* + 00**
	Std	1.30*E + *01	1.25*E + *02	1.97*E + *00	**0.00*E + *00**	**0.00*E* + 00**
	Rank	4	5	3	1	1

F6	Best	−**1.04*E + *01**	−6.43*E + *00	−**1.04*E + *01**	−**1.04*E + *01**	−**1.04*E* + 01**
	Worst	−2.75*E + *00	−5.28*E − *01	−5.09*E + *00	−5.09*E + *00	−**1.04*E* + 01**
	Ave	−8.59*E + *00	−1.76*E + *00	−9.87*E + *00	−9.34*E + *00	−**1.04*E* + 01**
	Std	3.11*E + *00	1.36*E + *00	1.62*E + *00	2.16*E + *00	**2.53E* − *07**
	Rank	4	5	2	3	1
Average rank		4	5	2.83	2	1

**Table 4:** CEC2017 test results.

	Index	PSO	DE	GWO	CS	MSSCS	SSA	GPSSA
F1	Ave	3.32*E + *03	3.44*E + *07	8.25*E + *08	9.97*E + *07	3.24*E + *03	3.82*E + *03	**1.57*E + *03**
	Std	3.40*E + *03	2.68*E + *06	5.83*E + *08	4.18*E + *07	3.35*E + *03	3.29*E + *03	**2.26*E + *03**
	Rank	3	5	7	6	2	4	1

F3	Ave	**3.00*E + *02**	1.22*E + *05	2.82*E + *04	3.81*E + *04	2.32*E + *04	5.03*E + *04	2.19*E + *04
	Std	**1.03*E − *01**	9.82*E + *03	9.91*E + *03	1.23*E + *04	7.21*E + *03	2.05*E + *04	1.47*E + *04
	Rank	1	7	4	5	3	6	2

F4	Ave	**4.73*E + *02**	5.41*E + *02	5.35*E + *02	5.12*E + *02	5.06*E + *02	5.10*E + *02	4.88*E + *02
	Std	2.77*E + *01	**4.18*E + *00**	2.72*E + *01	2.62*E + *01	2.28*E + *01	1.58*E + *01	2.90*E + *01
	Rank	1	7	6	5	3	4	2

F5	Ave	6.38*E + *02	6.82*E + *02	8.03*E + *02	6.33*E + *02	6.14*E + *02	7.80*E + *02	**5.95*E + *02**
	Std	1.30*E + *01	1.11*E + *01	**7.68*E + *00**	1.89*E + *01	1.79*E + *01	6.20*E + *01	3.72*E + *01
	Rank	4	5	7	3	2	6	1

F6	Ave	6.38*E + *02	**6.02*E + *02**	6.57*E + *02	6.25*E + *02	6.30*E + *02	6.65*E + *02	6.03*E + *02
	Std	9.06*E + *00	**1.06*E − *01**	6.18*E + *00	2.46*E − *01	1.66*E − *01	7.27*E + *00	1.55*E + *00
	Rank	5	1	6	3	4	7	2

F7	Ave	**8.30*E + *02**	9.28*E + *02	1.33*E + *03	8.64*E + *02	8.69*E + *02	1.33*E + *03	8.42*E + *02
	Std	2.13*E + *01	**7.59*E + *00**	1.01*E + *01	2.09*E + *01	1.96*E + *01	1.36*E + *01	2.72*E + *01
	Rank	1	5	7	3	4	6	2

F8	Ave	9.11*E + *02	9.85*E + *02	9.74*E + *02	9.47*E + *02	9.29*E + *02	9.91*E + *02	**8.86*E + *02**
	Std	1.58*E + *01	**9.28*E + *00**	3.22*E + *01	1.78*E + *01	1.66*E + *01	3.13*E + *01	2.55*E + *01
	Rank	2	6	5	4	3	7	1

F9	Ave	3.08*E + *03	2.89*E + *03	5.41*E + *03	1.05*E + *03	**1.00*E + *03**	5.42*E + *03	1.38*E + *03
	Std	5.67*E + *02	2.09*E + *02	**3.09*E + *01**	7.65*E + *01	5.66*E + *01	1.10*E + *02	3.09*E + *02
	Rank	5	4	6	2	1	7	3

F10	Ave	**4.23*E + *03**	7.21*E + *03	5.75*E + *03	5.41*E + *03	4.86*E + *03	6.25*E + *03	4.43*E + *03
	Std	5.71*E + *02	**1.93*E + *02**	1.02*E + *03	2.80*E + *02	4.16*E + *02	1.13*E + *03	1.12*E + *03
	Rank	1	7	5	4	3	6	2

F11	Ave	1.20*E + *03	1.62*E + *03	1.40*E + *03	1.21*E + *03	**1.20*E + *03**	1.24*E + *03	1.22*E + *03
	Std	**2.28*E + *01**	8.83*E + *01	9.95*E + *01	2.80*E + *01	2.62*E + *01	4.38*E + *01	4.74*E + *01
	Rank	2	7	6	3	1	5	4

F12	Ave	**5.18*E + *04**	5.16*E + *07	2.78*E + *07	8.08*E + *09	7.08*E + *09	1.92*E + *06	1.16*E + *06
	Std	**2.60*E + *04**	6.84*E + *06	2.74*E + *07	4.21*E + *09	4.93*E + *09	1.36*E + *06	1.50*E + *06
	Rank	1	5	4	7	6	3	2

F13	Ave	9.40*E + *03	4.28*E + *06	2.48*E + *06	7.07*E + *08	3.52*E + *08	1.49*E + *07	**4.56*E + *03**
	Std	1.14*E + *04	1.35*E + *06	1.31*E + *07	2.64*E + *09	1.92*E + *09	5.73*E + *07	**2.40*E + *03**
	Rank	2	4	3	7	6	5	1

F14	Ave	8.51*E + *03	1.17*E + *05	2.94*E + *05	1.59*E + *03	**1.56*E + *03**	1.76*E + *04	6.20*E + *03
	Std	4.65*E + *03	5.33*E + *04	3.29*E + *05	2.51*E + *01	**1.28*E + *01**	1.44*E + *04	1.18*E + *03
	Rank	4	6	7	2	1	5	3

F15	Ave	1.61*E + *04	3.74*E + *05	3.48*E + *04	2.15*E + *03	**1.73*E + *03**	7.62*E + *03	3.57*E + *03
	Std	1.19*E + *04	2.64*E + *05	2.32*E + *04	1.77*E + *02	**3.09*E + *01**	6.45*E + *03	7.42*E + *02
	Rank	5	7	6	2	1	4	3

F16	Ave	2.53*E + *03	2.74*E + *03	3.37*E + *03	2.51*E + *03	2.36*E + *03	3.57*E + *03	**2.36*E + *03**
	Std	1.82*E + *02	**8.27*E + *01**	5.91*E + *02	2.51*E + *02	2.05*E + *02	6.71*E + *02	2.63*E + *02
	Rank	4	5	6	3	2	7	1

F17	Ave	2.12*E + *03	2.01*E + *03	2.79*E + *03	1.98*E + *03	**1.96*E + *03**	2.87*E + *03	1.98*E + *03
	Std	2.07*E + *02	**5.48*E + *01**	2.84*E + *02	9.25*E + *01	6.33*E + *01	2.51*E + *02	1.73*E + *02
	Rank	5	4	6	2	1	7	3

F18	Ave	1.45*E + *05	1.21*E + *06	7.22*E + *05	1.17*E + *05	**5.71*E + *04**	1.25*E + *05	3.61*E + *05
	Std	1.47*E + *05	3.49*E + *05	6.37*E + *05	4.01*E + *04	**2.29*E + *04**	2.10*E + *05	1.63*E + *05
	Rank	4	7	6	2	1	3	5

F19	Ave	9.39*E + *03	4.08*E + *05	7.29*E + *05	2.84*E + *03	**2.08*E + *03**	6.35*E + *03	2.86*E + *03
	Std	1.02*E + *04	9.24*E + *04	2.38*E + *06	4.61*E + *02	**2.63*E + *01**	3.84*E + *03	5.71*E + *02
	Rank	5	6	7	2	1	4	3

F20	Ave	2.46*E + *03	2.34*E + *03	2.80*E + *03	2.32*E + *03	**2.30*E + *03**	2.72*E + *03	2.37*E + *03
	Std	1.18*E + *02	6.38*E + *01	**4.06*E + *01**	9.61*E + *01	8.90*E + *01	2.01*E + *02	1.13*E + *02
	Rank	5	3	7	2	1	6	4

F21	Ave	2.42*E + *03	2.49*E + *03	2.56*E + *03	2.49*E + *03	2.49*E + *03	2.55*E + *03	**2.38*E + *03**
	Std	2.25*E + *01	**7.43*E + *00**	2.71*E + *01	4.14*E + *01	4.97*E + *01	2.46*E + *01	2.20*E + *01
	Rank	2	3	7	5	4	6	1

F22	Ave	**3.46*E + *03**	4.51*E + *03	6.95*E + *03	3.60*E + *03	3.61*E + *03	6.97*E + *03	4.55*E + *03
	Std	1.85*E + *03	**2.43*E + *02**	1.76*E + *03	2.04*E + *03	1.86*E + *03	1.09*E + *03	2.28*E + *03
	Rank	1	4	6	2	3	7	5

F23	Ave	3.03*E + *03	2.83*E + *03	3.08*E + *03	2.85*E + *03	2.87*E + *03	3.26*E + *03	**2.79*E + *03**
	Std	9.38*E + *01	**7.69*E + *00**	8.69*E + *01	3.23*E + *01	2.04*E + *01	1.09*E + *02	7.37*E + *01
	Rank	5	2	6	3	4	7	1

F24	Ave	3.14*E + *03	3.02*E + *03	3.21*E + *03	3.02*E + *03	3.03*E + *03	3.39*E + *03	**2.91*E + *03**
	Std	1.06*E + *02	**6.89*E + *00**	5.94*E + *01	2.12*E + *01	6.03*E + *01	9.44*E + *01	3.89*E + *01
	Rank	5	2	6	3	4	7	1

F25	Ave	**2.88*E + *03**	2.92*E + *03	2.96*E + *03	3.00*E + *03	3.03*E + *03	2.91*E + *03	2.90*E + *03
	Std	8.15*E + *00	5.19*E + *00	2.40*E + *01	1.48*E + *00	**9.70*E − *01**	1.51*E + *01	1.85*E + *01
	Rank	1	4	5	6	7	3	2

F26	Ave	6.02*E + *03	5.40*E + *03	8.84*E + *03	3.49*E + *03	**3.37*E + *03**	7.63*E + *03	4.45*E + *03
	Std	2.17*E + *03	**8.24*E + *01**	9.26*E + *02	8.16*E + *02	6.27*E + *02	1.54*E + *03	3.63*E + *02
	Rank	5	4	7	2	1	6	3

F27	Ave	**3.21*E + *03**	3.23*E + *03	3.46*E + *03	3.34*E + *03	3.37*E + *03	3.59*E + *03	3.23*E + *03
	Std	1.05*E + *02	**3.01*E + *00**	1.17*E + *02	8.91*E + *00	1.01*E + *01	2.75*E + *02	1.86*E + *01
	Rank	1	3	6	4	5	7	2

F28	Ave	3.19*E + *03	3.33*E + *03	3.36*E + *03	3.36*E + *03	3.37*E + *03	3.24*E + *03	**3.19*E + *03**
	Std	5.53*E + *01	**6.87*E + *00**	3.59*E + *01	2.30*E + *01	2.13*E + *01	2.37*E + *01	5.41*E + *01
	Rank	2	4	6	5	7	3	1

F29	Ave	3.78*E + *03	4.03*E + *03	5.37*E + *03	3.78*E + *03	3.76*E + *03	5.02*E + *03	**3.68*E + *03**
	Std	2.43*E + *02	**9.67*E + *01**	9.24*E + *02	1.10*E + *02	1.18*E + *02	5.75*E + *02	1.42*E + *02
	Rank	3	5	7	4	2	6	1

F30	Ave	**5.26*E + *03**	5.28*E + *05	7.35*E + *06	2.41*E + *04	1.33*E + *04	2.76*E + *04	2.43*E + *04
	Std	**2.38*E + *03**	1.63*E + *05	3.03*E + *06	6.52*E + *03	3.18*E + *03	1.18*E + *04	1.02*E + *04
	Rank	1	6	7	3	2	5	4
Average rank	2.97	4.76	6.00	3.59	2.93	5.48	2.28	

**Table 5:** Wilcoxon rank-sum test results.

*F*	F1	F3	F4	F5	F6	F7	F8	F9	F10	F11
PSO	2.20*E − *02	2.78*E − *11	4.52*E − *01	1.15*E − *07	2.51*E − *11	6.71*E − *02	8.20*E − *07	3.25*E − *11	6.62*E − *01	7.18*E − *02
DE	2.66*E − *11	2.80*E − *11	7.74*E − *09	8.10*E − *09	2.39*E − *01	2.57*E − *11	2.38*E − *10	2.79*E − *11	7.22*E − *09	2.75*E − *11
GWO	2.69*E − *11	8.97*E − *03	1.90*E − *07	2.44*E − *11	2.51*E − *11	2.73*E − *11	1.63*E − *10	2.76*E − *11	2.10*E − *06	6.20*E − *10
CS	2.65*E − *11	8.15*E − *06	1.25*E − *04	5.09*E − *07	2.88*E − *11	2.99*E − *03	7.59*E − *10	3.02*E − *06	4.20*E − *08	6.30*E − *01
MSSCS	2.67*E − *02	1.58*E − *01	8.61*E − *04	3.33*E − *04	2.88*E − *11	1.14*E − *04	3.60*E − *09	5.75*E − *09	3.82*E − *03	7.21*E − *03
SSA	7.38*E − *03	1.74*E − *08	8.73*E − *05	9.22*E − *11	2.72*E − *11	2.52*E − *11	1.02*E − *10	2.66*E − *11	4.03*E − *08	3.02*E − *01

	F12	F13	F14	F15	F16	F17	F18	F19	F20	F21
PSO	2.94*E − *11	5.58*E − *01	5.28*E − *03	1.02*E − *03	3.72*E − *04	4.36*E − *03	2.21*E − *05	2.50*E − *01	1.06*E − *02	1.43*E − *08
DE	2.59*E − *11	2.83*E − *11	2.58*E − *11	2.42*E − *11	5.14*E − *09	7.93*E − *02	4.48*E − *11	2.57*E − *11	6.09*E − *01	7.48*E − *11
CS	6.16*E − *11	2.81*E − *11	3.99*E − *10	2.45*E − *11	2.00*E − *10	2.83*E − *11	6.43*E − *03	2.52*E − *11	2.42*E − *11	2.78*E − *11
MSSCS	2.23*E − *08	6.88*E − *09	2.63*E − *11	4.17*E − *11	1.83*E − *03	3.25*E − *01	1.42*E − *07	8.53*E − *01	1.90*E − *01	1.13*E − *09
GWO	1.40*E − *04	2.60*E − *03	2.63*E − *11	2.52*E − *11	6.84*E − *01	3.95*E − *01	8.08*E − *09	8.13*E − *10	4.34*E − *02	1.51*E − *08
SSA	3.08*E − *02	2.92*E − *09	3.06*E − *10	2.73*E − *05	1.60*E − *10	2.64*E − *11	5.30*E − *07	4.25*E − *04	3.80*E − *09	2.41*E − *11

	F22	F23	F24	F25	F26	F27	F28	F29	F30	+/ = /−
PSO	2.52*E − *04	2.74*E − *11	8.73*E − *11	1.06*E − *06	7.61*E − *03	9.31*E − *08	8.65*E − *01	1.44*E − *01	2.41*E − *11	21/0/8
DE	8.19*E − *01	1.85*E − *01	5.22*E − *10	2.94*E − *06	4.81*E − *10	9.70*E − *01	2.78*E − *11	3.07*E − *10	2.78*E − *11	23/0/6
GWO	2.96*E − *05	2.83*E − *11	2.78*E − *11	1.95*E − *09	2.43*E − *11	2.83*E − *11	3.74*E − *11	4.59*E − *11	2.75*E − *11	29/0/0
CS	2.91*E − *02	1.50*E − *02	7.03*E − *10	2.72*E − *11	3.05*E − *04	2.93*E − *11	3.00*E − *11	2.02*E − *03	1.53*E − *01	25/0/5
MSSCS	5.36*E − *02	1.59*E − *03	4.78*E − *09	2.72*E − *11	2.32*E − *06	2.93*E − *11	3.00*E − *11	7.44*E − *02	1.24*E − *09	25/0/5
SSA	6.79*E − *07	2.47*E − *11	2.48*E − *11	3.49*E − *03	4.63*E − *10	2.44*E − *11	9.40*E − *05	2.68*E − *11	1.66*E − *01	27/0/2

**Table 6:** UAV track planning results.

Index	PSO	DE	GWO	SSA	GPSSA
Best	80.8240	80.6203	80.8124	79.6252	**76.0988**
Worst	105.1887	104.2779	105.1887	107.1757	**89.3498**
Ave	88.6080	87.4127	86.4252	92.5325	**82.4084**
Std	9.1291	8.1642	7.9080	9.3197	**3.6872**

## Data Availability

The data used to support the findings of this study are available from the corresponding author upon request.
